# Manipulations of Oblique Pulling Affect Sacroiliac Joint Displacements and Ligament Strains: A Finite Element Analysis

**DOI:** 10.1155/2023/2840421

**Published:** 2023-01-03

**Authors:** Zhun Xu, Ziyu Feng, Zhaocong Zhang, Kunmu Zhang, Yikai Li

**Affiliations:** ^1^Department of Spine Surgery, The First Affiliated Hospital, Hengyang Medical School, University of South China, Hengyang 421000, Hunan Province, China; ^2^School of Traditional Chinese Medicine, Southern Medical University, No. 1838, Guangzhou Avenue North, Baiyun District, Guangzhou 510515, Guangdong Province, China; ^3^The Second Affiliated Hospital of Fujian University of Traditional Chinese Medicine, No. 282 Wusi Road, Gulou District, Fuzhou 350003, Fujian Province, China

## Abstract

**Objective:**

Clinical studies have found that manipulation of oblique pulling has a good clinical effect on sacroiliac joint pain. However, there is no uniform standard for manipulation of oblique pulling at present. The purpose of this study was to investigate the effects of four manipulations of oblique pulling on sacroiliac joint and surrounding ligaments.

**Methods:**

A three-dimensional finite element model of the pelvis was established. Four manipulations of oblique pulling were simulated. The stresses and displacements of sacroiliac joint and the strains of surrounding ligaments were analyzed under four manipulations of oblique pulling.

**Results:**

Manipulation of oblique pulling F2 and F3 caused the highest and lowest stress on the pelvis, at 85.0 and 52.6 MPa, respectively. Manipulation of oblique pulling F3 and F1 produced the highest and lowest stress on the left sacroiliac joint, at 6.6 and 5.6 MPa, respectively. The four manipulations of oblique pulling mainly produced anterior-posterior displacement. The maximum value was 1.21 mm, produced by manipulation of oblique pulling F2, while the minimal value was 0.96 mm, produced by manipulation of oblique pulling F3. The four manipulations of oblique pulling could all cause different degrees of ligament strain, and manipulation of oblique pulling F2 produced the greatest ligament strain.

**Conclusions:**

The four manipulations of oblique pulling all produced small displacements of sacroiliac joint. However, they produced different degrees of ligament strain. Manipulation of oblique pulling F2 produced the largest displacement of sacroiliac joint and the greatest ligament strain, which could provide a certain reference for physiotherapists.

## 1. Introduction

Lower back pain usually caused by lumbar diseases, including myofasciitis, lumbar disc herniation, and lumbar spondylolisthesis, is a common clinical symptom [1–3]. In recent years, it has been found that the lesion of sacroiliac joint (SIJ) can also cause lower back pain, accounting for 14.5%∼22.5% [4]. Commonly, abnormal gait, heavy physical exertion, leg length discrepancy, and scoliosis may be factors related to SIJ pain without specific causes. The mechanism may include the following processes: pathogenic factors acting on the auricular surface of the sacrum and ilium may cause injury to the ligaments or muscles around the SIJ, which will result in slight movement of the SIJ, making the joints difficult to reset. The mechanical environment of the joints may ultimately be imbalanced, and the soft tissues will be damaged. This condition is clinically referred to as SIJ subluxation [5].

There are many treatment methods for SIJ subluxation, mainly including the following: (1) take nonsteroidal anti-inflammatory drugs (NSAID) and drugs for promoting blood circulation, so as to achieve the effects of anti-inflammatory, and promote blood circulation and remove blood stasis [6, 7]. (2) Inject glucocorticoids into the SIJ via a guide wire to produce a direct anti-inflammatory effect [8–10]. (3) Pull the subluxated SIJ back to the normal position by manipulation to reduce nerve stimulation and relieve pain [11–14]. At present, the three methods have been applied in clinical treatment, and manipulation is the most widely used [15, 16].

Manipulation relieves the low back pain by changing the mechanical environment of SIJ and surrounding tissue. This treatment method has little side effects, and can be easily accepted by patients. A large number of clinical studies have shown that manipulation of oblique pulling (MOP) has a good effect on SIJ subluxation [17–19]. The detailed procedure are as follows: the patient is in the right decubitus position. The right lower extremity is straight, and the left lower extremity is slightly bent. The therapist stands at the patient's ventral side. The therapist holds the patient in position with one hand on the back of the sacrum, the other hand on the anterior-superior spine, pushing the ilium towards the back. However, the position and direction of the manipulative force varies from therapists. There is no uniform standard for MOP at present. Does MOP with different force points and directions produce different effects on the SIJ and its surrounding ligaments? None of these issues has been studied. Therefore, this study intends to establish a three-dimensional finite element model of the pelvis and explore the effects of MOP on the stress and displacement of SIJ and strain of the surrounding ligament by simulating four common MOPs.

## 2. Materials and Methods

### 2.1. Model Construction

A 3D finite element model of the pelvis was established. Three-dimensional models of the sacrum and ilia were reconstructed from the computed tomography (CT) images of a healthy male volunteer (34 years old, 170 cm in height, and 65 kg in weight) using Mimics 20.0 (Materialise Company, Leuven, Belgium), and the cortical and cancellous regions of the bones were distinguished. Axial slices 0.5 mm thick spanning the entire pelvis were selected for model construction. All surface models were meshed using Geomagic 2013 (Raindrop Company, Marble Hill, USA). The SIJ was composed of cartilage and the endplate of the sacrum and the ilia, with their surrounding ligaments. The cartilage was reconstructed with a uniform thickness. The regions of the articular surfaces were based on CT images, and the thicknesses of the cartilage were acquired from the literature [20]. The sacral and iliac cartilages had thicknesses of 2 mm and 1 mm, respectively. The bone endplate thicknesses of the sacral and iliac parts of the cartilage were assumed to be 0.23 mm and 0.36 mm, respectively. The gap between the two cartilages was set at 0.3 mm [20]. The material properties chosen from previous studies [20, 21] are summarized in Table 1.

The anterior sacroiliac ligament (ASL), short posterior sacroiliac ligament (SPSL), long posterior sacroiliac ligament (LPSL), sacrospinous ligament (SS), interosseous sacroiliac ligament (ISL), and sacrotuberous ligament (ST) complexes were modelled as 3D tension-only truss elements. The material properties of each ligament were obtained from the literature [21]. The attachment regions were chosen according to the literature [20]. In total, the pelvic model contained 458,867 elements and 201,982 nodes.  Figure 1 shows the intact model with ligamentous attachments.

### 2.2. Simulation of MOPs

The simulation of MOP was as follows: the magnitudes of the forces were determined by determining the manipulative power of five therapists using a biomechanical testing machine. The average manipulative force was 600 N [22]. Therefore, a large part of the sacrum and the right iliac crest were fixed. Then, a push force of 600 N along the ventral-dorsal direction was applied to the left anterior-superior spine or anterior-inferior iliac spine.

There were four MOPs. MOP-F1: the force was applied at the left anterior-inferior iliac spine in a direction of 30° from the sagittal plane which roughly paralleled to the SIJ surface. MOP-F2: the force was applied at the left anterior-inferior iliac spine, parallel to the sagittal plane. MOP-F3: the force was applied at the left anterior-superior iliac spine in a direction of 30° from the SIJ surface. MOP-F4: the force was applied at the left anterior-superior iliac spine, parallel to the sagittal plane. The detailed loading and boundary conditions, as well as the *x*-, *y*-, and *z*-axes, are described in Figure 2. The compressive stresses and displacements of SIJ and the strains of ligaments for four MOPs were then investigated using Abaqus 2018 (Dassault Syst*è*mes S. A Company, Massachusetts, USA).

### 2.3. Mesh Convergence Study

In order to evaluate the degree of accuracy of the pelvic model, the mesh convergence study was carried out. Four mesh models were established according to different mesh fineness. The number of elements and nodes in each model are shown in Table 2. Following boundary conditions and material properties, loads, and constraints were described in detail in the abovementioned sections. MOP-F1, F2, F3, and F4 were applied to these meshes. Finally, the maximum stresses and displacements of the four models on the left SIJ surface of the sacrum under four MOPs were analyzed.

### 2.4. Model Validation

Two studies were performed to validate this model. For the pelvic model, the distribution of the main strain of the pelvis was compared with that reported in the study of Zhang et al. [23]. In our model, the distribution of the main strain of the pelvis was analyzed under the single-legged stance. For the sacrum model, the relationship between displacement and load was compared with that indicated in cadaveric [24] and computational studies [20, 25]. When the bilateral ilia were fixed, five translational forces (anterior, posterior, superior, inferior, and mediolateral) of 294 N and three moments (flexion, extension, and axial rotation) of 42 Nm were applied to the centre of the sacrum, respectively. The displacements of a node lying in the midsagittal plane between the inferior S1 and superior S2 vertebral endplates were calculated. In this model, the displacements were investigated under the same loading.

## 3. Results

### 3.1. Mesh Convergence Study

The maximum stress and maximum displacement on the left SIJ surface of the sacrum were analyzed for each of the meshes, under MOP-F1, F2, F3, and F4, which are shown in Figure 3. The differences in maximum stress and maximum displacement between mesh 3 and mesh 4 under four MOPs were less than 5%, which was considered as reasonably close ranges. According to these results, mesh 3 with 458,867 elements was selected for further study.

### 3.2. Model Validation

The stresses were located mainly in the upper and posterior areas of the acetabulum and extended to the iliac crest, the incisura ischiadica major, and the rear acetabulum. The area of stress concentration and maximum value of stress were consistent with those reported in a previous study [23]. Under eight loading conditions, the displacements agreed not only with those in an experimental study but also with those in some computational studies [20, 24, 25], and these results are shown in Figure 4.

### 3.3. Stress of the Pelvis and SIJ

The stress distributions of the pelvis under four MOPs are shown in Figure 5. Under MOP-F1, the stress of the ventral pelvis was mainly concentrated on the left SIJ, extended to the arcuate line, the right SIJ, the right anterior-inferior iliac spine, the upper part of the right acetabulum, and the outer upper edge of the right pubis. While the stress of the dorsal pelvis was mainly concentrated around the left posterior inferior iliac spine and the greater ischial notch. The maximum stress value was 76.9 MPa. Under MOP-F2, the area of stress concentration was roughly the same as that under MOP-F1, but the maximum stress value was higher, at 85.0 MPa. Under MOP-F3, the stress of the ventral pelvis was mainly concentrated on the left iliac crest, the left SIJ, the arcuate line, and the superior ramus of the pubis, while the stress of the dorsal pelvis was mainly concentrated on the left iliac crest and the greater sciatic notch. The maximum stress value was 52.6 MPa. Under MOP-F4, the area of stress concentration was roughly the same as that under MOP-F3. The maximum stress value was 80.0 MPa.

The distributions of stresses on the SIJ surface of the sacrum are shown in Figure 6. Under four MOPs, the principal stresses were concentrated on the anterior and inferior part of the left SIJ. Higher stress was observed on the left SIJ for the four MOPs. Among them, MOP-F3 produced the highest stress on the left SIJ, at 6.6 MPa, while MOP-F1 produced the lowest stress on the left SIJ, at 5.6 MPa.

### 3.4. Displacement of SIJ

In MOP-F1, the displacements of the left SIJ were 1.088, 0.305, and 0.033 mm in the anterior-posterior (AP), superior-inferior (SI) and medial-lateral (MI) direction, respectively. In MOP-F2, the displacements were 1.211, 0.186, and 0.064 mm in the AP, SI, and MI direction, respectively. In MOP-F3, the displacements were 0.962, 0.048, and 0.117 mm in the AP, SI, and MI direction, respectively. In MOP-F4, the displacements were 1.105, 0.064, and 0.094 mm in the AP, SI, and MI direction, respectively. The four MOPs mainly produced anterior-posterior displacement. The displacement of the left SIJ under four MOPs are shown in Figure 7.

### 3.5. Strain of Ligaments

The strains of six ligaments under four MOPs are shown in Figure 8. For most of the ligaments, the strain of the left ligament was greater than that of the right ligament under four MOPs. In MOP-F1, the left SS, ASL, and ISL had a higher strain value, which were 3.71, 1.41, and 1.36%, respectively. In MOP-F2, the left SS, ST, and ASL had a higher strain value, which were 4.29, 1.51, and 1.28%, respectively. In MOP-F3, the left SS, ASL, and ST had a higher strain value, which were 3.05, 1.61, and 1.09%, respectively. In MOP-F4, the left SS, SPSL, and ASL had a higher strain value, which were 2.85, 1.90, and 1.04%, respectively.

## 4. Discussion

SIJ subluxation is a common clinical disease [26, 27]. The main cause of the disease is the minor displacement of SIJ or the injury of surrounding ligaments. According to many clinical reports [17, 28, 29], MOP could achieve good results in the treatment of SIJ subluxation. However, MOP has had no uniform standard for force point and direction. In this study, we established a three-dimensional finite element model of the pelvis to explore the effects of MOP with different force points and directions on SIJ.

MOP-F1 and F2 were applied at the anterior-inferior iliac spine, while MOP-F3 and F4 were applied at the anterior-superior iliac spine. The force direction of F1 and F3 were roughly parallel to the SIJ surface, and the force direction of F2 and F4 were parallel to the sagittal plane of the pelvis. Anatomically, the anterior-inferior iliac spine is located inside and below the anterior-superior iliac spine, closer to the SIJ surface. Therefore, under the same direction of manipulation, MOP-F1 and F2 could produce greater maximum stress on the left hemi-pelvis than MOP-F3 and F4. In addition, since the anterior-superior iliac spine was closer to the iliac crest region, MOP-F3 and F4 also caused greater stress on the left iliac crest region than MOP-F1 and F2. From the perspective of the mechanical mechanism, the direction of manipulation parallel to the sagittal plane is more likely to produce greater stress on the left hemi-pelvis than that parallel to the SIJ surface. Furthermore, the torque on the right hemi-pelvis was also greater, which could lead to greater stress on the right hemi-pelvis. Therefore, MOP-F2 and F4 produced greater stress on the left and right pelvis than MOP-F1 and F3.

The lower 1/3 part of SIJ is the synovial joint, and the posterior and upper 1/3 part of SIJ is connected by the interosseous ligaments [30], so the motion of SIJ is mainly undertaken by the lower 1/3 part of SIJ. The stresses on SIJ surfaces of the sacra produced by four MOPs mainly distributed in the front and lower part of SIJ surfaces, which was related to the anatomical structure of SIJ. Due to the force point located on the left pelvis, the greater stresses were observed on the left SIJ surfaces under four MOPs. Compared with MOP-F2, MOP-F1 produced a smaller maximum stress on the left SIJ surface, which was connected to the direction of MOP-F1 parallel to the SIJ surface. Compared with MOP-F4, MOP-F3 produced a greater maximum stress on the left SIJ surface. This phenomenon suggested that the SIJ surface was compressed and the motion forms of SIJ included translation and rotation.

The displacement of the left SIJ was greater than that of the right side under four MOPs. The displacement of the left SIJ was 0.96∼1.21 mm in AP direction, 0.03∼0.12 mm in MI direction, and 0.05∼0.31 mm in SI direction. The values were all within 3 mm, which was consistent with previous research results [31, 32]. Under four MOPs, the displacement in the AP direction was the largest in the three directions, which might be related to the fact that MOP could turn the pelvis outward. In the AP direction, MOP-F2 and F4 produced the largest displacement of the left SIJ. The directions of forces applied by MOP-F2 and F4 were parallel to the sagittal plane, which was more likely to cause SIJ movement in the AP direction than the directions of the force parallel to the SIJ surface. In the MI direction, MOP-F3 and F4 produced the largest displacements. The force points of the two manipulations were at the anterior-superior iliac spine, which were far from the SIJ surface. Thus, the force arm was longer, which was easier to produce displacement in the MI direction. The sacrum is broad at the top and narrow at the bottom. It is wedge-shaped and lies between the iliac bones on both sides forming SIJ [33]. This special structure makes the SIJ move up easily, but move down difficultly. The anterior-inferior iliac spine is located inside and below the anterior-superior iliac spine. Thus, MOP-F1 and F2 applied at the anterior-inferior iliac spine could produce a larger upward displacement in the SI direction.

Ligaments play an important role in maintaining pelvis stability. Abdelfattah and Moed [34] found that the pubic symphysis and the anterior sacroiliac ligament played a key part in maintaining pelvis stability when the pelvis suffered “book-turning” violence. Sichting et al. [35] considered that the ligaments around SIJ not only played a role in maintaining mechanical stability of SIJ, but also acted as a neuromuscular feedback mechanism. Eichenseer et al. [25] through a finite element model, demonstrated that with the decrease of ligament stiffness, the stress and movement of SIJ would increase. Bohme et al. [36] found that the anterior sacroiliac ligament and the sacrotuberous ligament bore the largest load in the case of anterior and posterior compression fractures of the pelvis, accounting for 80% and 17% of the total load, respectively. The sacrospinous ligament played an important role in maintaining vertical stability of the pelvis. Our results indicated that the strains of the sacrospinous ligament, the anterior sacroiliac ligament, and the interosseous ligament were larger than the other three ligaments in most cases under four MOPs. Among them, the strain of sacrospinous ligament caused by MOP-F2 was the largest, at 4.29%. Under MOP-F2, the displacement of SIJ was the largest, which led to the largest ligament strain. The anterior sacroiliac ligament is a broad and thin ligament located in the front of SIJ. The main displacement under four MOPs was in the AP direction, so the anterior sacroiliac ligament would produce a greater strain.

In this study, there were four types of MOP. MOP-F2 and F4 produced the larger displacement in the AP direction, at 1.21 and 1.11 mm, respectively. It showed that the manipulation parallel to the sagittal plane could cause a larger displacement. In addition, MOP-F2 and F4 also caused greater ligament strains. It could be seen that MOP-F2 and F4 are more effective manipulations to cause the displacement of SIJ and the strain of the surrounding ligaments.

There are some limitations in this study. First, the finite element model was established based on a single individual, while there are individual differences on age and gender for SIJ. Second, the ligaments in this model were built with linear materials, which had certain influence on reflecting the strain of ligaments. Third, this pelvic model only contained bones and ligaments. Soft tissues such as muscles and the skin were not considered. Fourth, manipulations were analyzed based on a normal SIJ in this model, but manipulations were applied to the subluxated SIJ clinically, so the results could not fully reflect the biomechanical characteristics of manipulations. Perhaps the diseased SIJ was less stable and easier to reduce under manipulation. The establishment of the finite element model of SIJ subluxation will benefit the further study of the disease.

## 5. Conclusions

In this study, a three-dimensional finite element model of the pelvis was established, and four manipulations with different force points and different directions were studied. The results showed that MOP-F3 and F4 caused greater stresses on the SIJ surface. The four MOPs all produced small displacements of the SIJ and different degrees of ligament strain. Among them, MOP-F2 and F4 could produce greater displacements of SIJ and ligament strains. MOP-F1 and F2 applied on the anterior-inferior iliac spine mainly produced the displacement in AP and SI directions, while F3 and F4 applied on the anterior-superior iliac spine mainly produced the displacement in AP and MI directions.

## Figures and Tables

**Figure 1:** Ventral (a) and dorsal (b) views of the finite element model. Ligaments are represented in color lines, with red arrows identifying each ligament complex (note the interosseous sacroiliac ligament is not visible in anterior-posterior views). ASL indicates anterior sacroiliac ligament; LPSL, long posterior sacroiliac ligament; SPSL, short posterior sacroiliac ligament; SS, sacrospinous ligament; ST, sacrotuberous ligament.

**Figure 2:** Loading and boundary conditions for four manipulations of oblique pulling. The yellow triangles represent the fixed sites of the pelvic model. The superior view (a, b, c, and d) and frontal view (e, f, g, and h) of the pelvis are shown, (a) and (e) manipulation of oblique pulling-F1; (b) and (f) manipulation of oblique pulling-F2; (c) and (g) manipulation of oblique pulling-F3; (d) and (h) manipulation of oblique pulling-F4.

**Figure 3:** (a) Maximum stresses on the left SIJ surface of the sacrum for different number of mesh elements, under MOP-F1, F2, F3, and F4. (b) Maximum displacements on the left SIJ surface of the sacrum for different number of mesh elements, under MOP-F1, F2, F3, and F4.

**Figure 4:** Comparison of sacral displacements under eight loadings comparable to those in previous experimental and computational studies.

**Figure 5:** Distribution of compressive stresses on the cortical bone of the pelvis under MOP-F1, F2, F3, and F4. The images of the local view are enlarged images in the red box of the general view.

**Figure 6:** Distribution of compressive stresses on the SIJ surface of the sacrum under MOP-F1, F2, F3, and F4.

**Figure 7:** The displacements of the left SIJ under MOP-F1, F2, F3, and F4. AP: anterior-posterior direction; SI: superior-inferior direction; MI: medial-lateral direction.

**Figure 8:** Ligament strains under MOP-F1, F2, F3, and F4. L: left; R: right; ASL: anterior sacroiliac ligament; ISL: interosseous sacroiliac ligament; SS: sacrospinous ligament; ST: sacrotuberous ligament; LPSL: long posterior sacroiliac ligament; SPSL: short posterior sacroiliac ligament.

**Table 1:** Material properties of the sacrum, ilium, pubic symphysis, and endplate.

		Young's modulus (MPa)	Poisson's ratio
Sacrum	Cortical	12,000	0.3
	Cancellous	100	0.2

Ilium	Cortical	12,000	0.3
	Cancellous	100	0.2

Pubic symphysis		5	0.45

Articular cartilage		100	0.3

Endplate		1000	0.4

**Table 2:** Element and node numbers for four different mesh resolutions.

	Element number	Node number
Mesh 1	142,007	58,480
Mesh 2	243,492	101,724
Mesh 3	458,867	201,982
Mesh 4	1,051,834	481,435

## Data Availability

The data used to support the findings of this study are available from the corresponding authors upon request.
